This article has been retracted.

# Application of Health Education Based on Phased Transition Theory Model in Continuous Nursing for Patients with Inflammatory Bowel Disease

**DOI:** 10.1155/2022/4194178

**Published:** 2022-07-09

**Authors:** Hongmei Xiao, Jun Ye

**Affiliations:** ^1^Department of Gastroenterology, Taizhou People's Hospital, Taizhou 225300, Jiangsu, China; ^2^Department of Nosocomial Infection Management, Jinhua People's Hospital, Jinhua 321015, Zhejiang, China

## Abstract

**Objective:**

To explore the application effect of health education based on phased transition theory model in the continuous nursing for patients with inflammatory bowel disease (IBD).

**Method:**

A total of 106 patients with IBD admitted to the hospital were enrolled as the research objects between October 2020 and September 2021. According to random number table method, they were divided into observation group and control group, 53 cases in each group. The control group was given routine nursing, while observation group was additionally given health education based on phased transition theory model. The nutritional status (serum prealbumin (PA), albumin (ALB), body mass index (BMI)), scores of Disease Knowledge Mastery Scale, exercise of self-care agency scale (ESCA), and Inflammatory Bowel Disease Questionnaire (IBDQ) were compared between the two groups before and after intervention.

**Results:**

After intervention, PA, ALB, and BMI in observation group were higher than those in control group (*P* < 0.05), scores of Disease Knowledge Mastery Scale, total mastery rate, scores and total score of ESCA, and scores and total score of IBDQ were significantly higher than those in control group (*P* < 0.05).

**Conclusion:**

The application of health education based on phased transformation theory model in the continuous nursing improves disease knowledge mastery, self-care ability, nutritional status, and quality of life in IBD patients.

## 1. Introduction

Inflammatory bowel disease (IBD) is a common chronic intestinal inflammatory disease, including ulcerative colitis and Crohn's disease. The main clinical manifestations of the patients are abdominal pain, diarrhea, and bloody stool [1–3]. IBD is characterized by a long course of disease, prolonged unhealing period, and a high recurrence rate. The treatment of IBD is difficult, and the patient's treatment compliance, dietary habits, and self-management ability can all have an important impact on treatment and recurrence [4]. Some studies have pointed out [5] that self-care and lifestyle of IBD patients after discharge are of great effect to improve the treatment outcome of patients, which is conducive to improving the quality of life and prognosis of patients. However, some patients lack the awareness of continuous care after discharge, which makes them poor in self-care ability and control of the disease. The phased transition theoretical model is a method that focuses on the process and needs of human behavior change, which can help to change the unhealthy behavior of patients and promote the development of their healthy behavior [6]. This theoretical model has been proved to have good effects in healthy education and nursing of chronic diseases such as asthma and diabetic nephropathy [7]. However, the value of its combination with continuous care in the clinical care of IBD patients is unclear. This study mainly explores the effect of the health education program based on the staged transition theoretical model in the continuation of care for IBD patients, to provide a theoretical basis for finding ways to improve self-care ability and quality of life in IBD patients.

## 2. Material and Methods

### 2.1. Clinical Data

106 inpatients with IBD who were admitted to our hospital from November 2020 to October 2021 were selected as the research subjects. According to the random number table method and random numbers generated by a computer, the patients were randomly divided into observation group and control group, with 53 patients in each group. Inclusion criteria: ① patients with age ≥18 years old and meeting the diagnostic criteria of IBD [8, 9]; ② the first onset, with complete clinical data; and ③ who are mentally and cognitively normal. Exclusion criteria: ① patients with language barrier, unable to communicate; ② with intestinal cancer or other malignant tumors; ③ with organic brain lesions and severe liver and kidney dysfunction; ④ who are unable to review and receive follow-up on time. This study was approved by the Medical Ethics Committee, and all subjects were informed and voluntarily participated in the study. There was no significant difference in baseline data such as age, gender, type of IBD, and years of education between the two groups (*P* > 0.05), as shown in Table 1.

### 2.2. Methods

The patients in the control group were given routine nursing care, which mainly included health education such as IBD-related knowledge lectures and watching IBD propaganda films to enhance the patients' cognition of the disease and recovery and to provide necessary psychological counseling, environmental care and dietary guidance, etc. Nursing staff urge patients to follow the doctor's orders to take medicines, give hospitalization guidance before discharge, instruct patients to seek medical treatment in time if they have problems, review them on time, and do not carry out any nursing intervention after discharge. We followed up by phone only and notified the patient to review regularly, the follow-up period was 2 months.

Based on the control group, the observation group adopted the health education program based on the theoretical model of phased transformation for continuous nursing. The specific methods are as follows: establishing a staged transformation theory model propaganda team, including 2 physicians, 2 nurses, 1 psychological counselor and 1 nutritionist in the gastroenterology department; learning the theory of staged transition and professional knowledge of postoperative care of IBD; after communicating with the patient, according to the patient's behavior and psychological characteristics, and combining the patient's needs, the continuous nursing work is divided into the following five stages: (1) preintention stage: at this stage, some patients have not yet realized the significance of IBD knowledge, self-care, and complication prevention to IBD. The total score of the scale is 100 points. Patients with a score of fewer than 70 points are included in the key health education goals, and patients with a score of 70 points and above are given normal education. The nursing staff invite relevant medical and nursing experts to hold knowledge lectures, watch videos, etc., to train patients on the mechanism of IBD, dietary precautions, self-care methods, prevention of complications, etc., and inform patients of the importance of following the doctor's prescription for medication in the chronic persistent period of the disease. Focus on educating patients to carry out analysis meetings, informing patients of assessment results and urging them to improve their health awareness. The intervention time is 1 week. (2) Intention stage: in this stage, patients already have a hospital that promotes the formation of healthy behaviors, but no definite plan has been produced. Nursing staff communicate and analyze with patients to find solutions for their current adverse health behaviors and their own health needs. Introduce the key content of health education to patients: instruct patients to evaluate the degree, nature, and location of their abdominal pain, record the nature and frequency of stool during diarrhea, analyze whether there are inducing factors, instruct patients to take targeted medication for relief, and return to the hospital for treatment if necessary. Help patients understand possible complications and corresponding treatment methods, teach patients how to clean the anus correctly, and prevent infection. In terms of medication, the importance of taking medication as prescribed by the doctor is emphasized to patients, the patients and their families are instructed the correct medication method, and the possible adverse reactions and treatment methods are explained. In terms of diet, guide patients to standardize their diet, eat more easily digestible, high-protein, and vitamin-rich foods and avoid fried and spicy foods. In life, guide patients to work and rest regularly, do physical exercise appropriately, and encourage patients to write a health diary. The intervention period was 1 week. (3) Preparation stage: comprehensively assess the patient's psychology, cognition, and condition, formulate clear goals and individualized health behavior promotion plans for the patient's current problems and disease characteristics, and sign a written agreement. Select the positive and negative cases of previous departments to share and provide personalized guidance according to the patient's psychological state and behavioral habits, to improve the patient's treatment and nursing compliance. A “rehabilitation nursing group” was established on the WeChat platform, and nursing staff continued to regularly push 1 piece of health education knowledge every day to improve health awareness. The intervention time was 2 weeks. (4) Action stage: according to the formulated care plan, nurses conduct regular telephone visits and home follow-ups to find out whether the patient is following the continuous care plan. Assess the patient's current cognition and condition, and adjust the plan in time; understand the patient's medication compliance, give guidance on time, make a family visit one month after discharge, urge the patient to adhere to regular and on-time medication, and regularly visit the hospital for follow-up visits. Adjust the medication under the guidance of the doctor, emphasizing the significance of the medication and the possible consequences of noncompliance. The intervention period was 2 weeks. (5) Maintenance stage: at this stage, the patient's self-care behavior has changed, but the speed of change may slow down over time, making it difficult to maintain. At this stage, strengthen the encouragement of patients, encourage and praise patients who have completed the plan well, and guide them to consolidate and maintain established healthy behaviors; those who do not complete the plan help them find problems and provide targeted guidance to help them solve problems, and appropriate psychological support is needed to strengthen their confidence in overcoming the disease and self-management, the intervention time was 2 weeks. The intervention time of the observation group was 8 weeks.

### 2.3. Observation Indicators

#### 2.3.1. Disease Knowledge Mastery

Before and after the intervention, the patient's disease knowledge mastery was evaluated by the self-made “IBD Disease Knowledge Mastery Scale.” The scale includes 4 items of IBD occurrence mechanism, common incentives, and complication prevention and daily nursing measures, with a total score of 100 points. Scores <70 points are not mastered, 70 points ≤ scores ≤90 points are partially mastered, and >90 points are fully mastered. The number of patients with complete and partial mastery of disease knowledge in the two groups after the intervention was counted, and the total mastery rate was calculated.

#### 2.3.2. Nutritional Status Indicators

Before and after the intervention, the body weight and height of the patients on an empty stomach in the morning were measured on-site with a height scale, and the body mass index (BMI) value was calculated. BMI = weight (kg)/height 2 (m2); and fasting cubital venous blood was collected from patients in the morning, and Hitachi 7180 automatic biochemical analyzer was used to detect albumin (Alb) and prealbumin (PA) level of the patients.

#### 2.3.3. Self-Care Ability

Before and after the intervention, the self-care ability assessment (ESCA) was used to evaluate the self-care ability of patients before and after nursing, including self-responsibility (6 items), self-care skills (12 items), health knowledge level (17 items), and self-concept (8 items), and the scores for each item are 24, 48, 68, and 32, respectively [10]. The higher the score indicates the better the patient's self-care ability.

#### 2.3.4. Evaluation of Patients' Quality of Life

Before and after the intervention, the Chinese version of the Inflammatory Bowel Disease Quality of Life Questionnaire [11] (IBDQ) was used to investigate the quality of life of the two groups of patients. The IBDQ includes four aspects: intestinal symptoms, systemic symptoms, emotional ability, and social ability. It is divided into 10, 5, 12, and 5 items. Each item is scored on a 7-point scale (1–7 points), with a total score of 224 points. A higher IBDQ score means the higher life quality of the patients.

### 2.4. Statistical Analysis

SPSS21.0 statistical software was used to analyze the experimental data, the count index was expressed as %, and the *χ*^2^ test was performed; the measurement indexes such as PA and ALB were expressed as “mean ± standard deviation ($\bar{X}\pm S$)”, and the *t*-test was conducted. *P* < 0.05 was considered statistically significant.

## 3. Results

### 3.1. Comparison of Disease Knowledge in the Two Groups before and after Intervention

After the intervention, the scores of disease knowledge mastery of the two groups of patients were significantly higher than those before the intervention (*P* < 0.05), and the disease knowledge mastery score and total mastery rate of the observation group were significantly higher than those of the control group (*P* < 0.05), as shown in Table 2.

### 3.2. Comparison of Nutritional Status Indicators in the Two Groups before and after Intervention

After the intervention, the levels of PA, ALB, and BMI in the two groups were lower than those before the intervention (*P* < 0.05); and the levels of PA, ALB, and BMI in the observation group were lower than those in the control group (*P* < 0.05), as shown in Table 3.

### 3.3. Comparison of Self-Care Ability of the Two Groups before and after the Intervention

After the intervention, the ESCA dimension scores and total scores in the two groups were higher than those before the intervention (*P* < 0.05); and the ESCA dimension scores and total scores in the observation group were higher than those in the control group (*P* < 0.05), as shown in Table 4.

### 3.4. Comparison of Quality of Life before and after Intervention between the Two Groups

After intervention, the scores and total scores of each dimension of IBDQ in the two groups were significantly higher than those before intervention (*P* < 0.05); and the scores and total scores of each dimension of IBDQ in the observation group were significantly higher than those in the control group (*P* < 0.05), as shown in Table 5.

## 4. Discussion

IBD is characterized by long course and prone to recurrence. The incidence of IBD is related to poor eating habits, anxiety, and depression. The clinical treatment of IBD is mainly by drug therapy, however the course of treatment is long and the compliance of some patients is poor, which leads to the relapse of IBD, is difficult to cure, and greatly reduces the quality of life of patients. However, IBD patients can still control the disease well and reduce recurrence by controlling diet, regulating emotions, and actively taking drugs. Studies have shown that [12] IBD patients formulate a reasonable care plan and program through continuous care, which can help patients obtain uninterrupted continuous care after discharge, improve their quality of life and treatment, and reduce the recurrence rate of the disease. The theoretical model of staged transition was proposed by the psychologist Prochaska, which mainly divides the process of human behavior change into five different stages, such as the unintentional period and the intentional period, which can promote the development of individual healthy behaviors [13, 14]. The combination of health education and continuous nursing based on the theoretical model of stage transition is conducive to the smooth implementation of continuous nursing measures, and it has been pointed out that it has a good intervention effect in the management of chronic diseases.

This study attempts to apply the health education program based on the staged transition theoretical model to the continued care of IBD patients. The results showed that after the intervention, the PA, ALB levels, and BMI of the patients in the observation group higher than those in the control group were significantly higher than those in the control group. It can be seen that this nursing model has significantly improved the patient's disease knowledge and self-care ability and improved the patient's nutritional status and quality of life. The health education program guided by the theoretical model of staged transformation in this study divides the transformation of patients' health behaviors into different stages and formulates targeted change plans according to the problems and unhealthy behaviors faced by the patients. In the process of implementing the patient plan, this nursing model provides key education and supervision to patients with insufficient cognition to improve their health awareness by assessing the degree of disease knowledge and cognition of patients; by training patients on the mechanism of IBD, dietary precautions, self-care methods, prevention of complications, etc., the importance of adhering to the doctor's prescription for medication is taught to patients, so that patients' disease knowledge and treatment compliance can be improved, which is helpful for patients after discharge [15]. IBD patients are prone to malnutrition, and in the absence of dietary guidance, patients are often confused by food choices. The dietary guidance of patients in the health education program based on the staged transition theoretical model can help patients eat healthy, improve their nutritional status, and reduce the occurrence of malnutrition [16].

In this study, the application of the health education program based on the theoretical model of staged transformation in the continuous nursing of patients with inflammatory bowel disease is based on the formulated targeted nursing plan, allowing patients to continue to receive continuous nursing at the level of nursing during hospitalization after discharge. Through staged behavioral intervention, the patients' awareness of active participation was improved, and they actively cooperated with the nursing plan to enhance their sense of self-responsibility and self-protection behavior; at the same time, this nursing model enables patients to master IBD-related health knowledge through staged and multichannel health education, pays attention to the adjustment of diet and lifestyle, changes unhealthy lifestyles and is conducive to disease control. After educating patients, patients have improved their self-management and nursing abilities through multiple follow-up visits, and they have guided and checked the changes in patients' health behaviors such as medication and living habits and cultivated patients' behaviors to comply with doctor's orders. After the patient's good living habits are consolidated during the maintenance period, they can promote the formation and maintenance of healthy behaviors and help improve the patient's physical health and quality of life [17].

In summary, the application of the health education program based on the staged transformation theoretical model in the continuous care of IBD patients improves the patients' disease knowledge and self-care ability and improves the nutritional status and quality of life of the patients.

## Figures and Tables

**Table 1:** Comparison of baseline data of two groups of patients.

Group	Gender (number of cases)		Age (year)	Education (year)	IBD type (number of cases)	
	Male	Female			Ulcerative colitis	Crohn's disease
Observation group (*n* = 53)	29	24	36.55 ± 4.88	11.25 ± 2.66	31	22
Control group (*n* = 53)	33	20	36.96 ± 6.50	11.17 ± 2.04	34	19
*χ* ^2^/*t*	0.622		0.372	0.164	0.358	
*P* value	0.430		0.711	0.870	0.550	

**Table 2:** Comparison of the mastery of disease knowledge between the two groups of patients.

Group	Overall mastery rate after intervention (number of cases (%))	Disease knowledge mastery score	
		Before intervention	After intervention
Observation group (*n* = 53)	50 (94.34)	66.35 ± 2.80	84.25 ± 4.29
Control group (*n* = 53)	41 (77.36)	66.91 ± 4.97	72.40 ± 3.40
*χ* ^2^/*t*	6.290	0.481	15.767
*P* value	0.012	0.632	0.000

**Table 3:** Comparison of BMI, PA, and ALB levels between the two groups before and after intervention (±*s*).

Group	PA (mg/L)		ALB (g/L)		BMI (kg/m^2^)	
	Before intervention	After intervention	Before intervention	After intervention	Before intervention	After intervention
Observation group (*n* = 53)	175.18 ± 12.22	213.34 ± 18.68^*∗*^	31.47 ± 3.46	32.07 ± 3.48^*∗*^	20.57 ± 1.15	20.87 ± 1.39^*∗*^
Control group (*n* = 53)	175.89 ± 11.88	257.23 ± 15.99^*∗*^	31.12 ± 2.20	34.34 ± 3.00	20.30 ± 1.08	22.86 ± 1.65
*t*	0.303	12.995	0.627	3.592	1.264	6.731
*P* value	0.762	0.000	0.533	0.001	0.209	0.000

*Note.* PA: serum prealbumin; ALB: albumin; BMI: body mass index; compared with the group of before intervention, ^*∗*^*P* < 0.05.

**Table 4:** Comparison of ESCA scores between the two groups before and after intervention (points, ±*s*).

Group	Self-responsibility		Mastery of health knowledge		Self-care skills		Self-concept		Total score	
	Before intervention	After intervention	Before intervention	After intervention	Before intervention	After intervention	Before intervention	After intervention	Before intervention	After intervention
Observation group (*n* = 53)	15.53 ± 2.33	21.40 ± 2.32^*∗*^	30.62 ± 3.46	57.30 ± 3.77^*∗*^	24.34 ± 3.11	35.00 ± 3.61^*∗*^	17.62 ± 2.40	28.42 ± 3.69^*∗*^	88.11 ± 5.91	142.11 ± 6.07^*∗*^
Control group (*n* = 53)	16.19 ± 2.10	17.92 ± 2.98^*∗*^	30.36 ± 2.96	45.60 ± 3.18^*∗*^	23.70 ± 2.28	28.25 ± 2.62^*∗*^	18.09 ± 2.70	21.26 ± 2.22^*∗*^	88.34 ± 4.45	113.04 ± 5.20^*∗*^
*t*	1.533	6.689	0.422	17.288	1.197	11.039	0.952	12.096	0.223	26.494
*P* value	0.128	0.000	0.674	0.000	0.234	0.000	0.343	0.000	0.824	0.000

*Note.* Compared with the group of before intervention, ^*∗*^*P* < 0.05.

**Table 5:** Comparison of IBDQ scores between the two groups before and after intervention (points, ±*s*).

Group	Intestinal symptoms		Systemic symptoms		Emotional capacity		Social competence		Total score	
	Before intervention	After intervention	Before intervention	After intervention	Before intervention	After intervention	Before intervention	After intervention	Before intervention	After intervention
Observation group (*n* = 53)	33.58 ± 3.52	53.51 ± 2.93^*∗*^	22.81 ± 2.42	33.55 ± 2.50^*∗*^	57.40 ± 4.21	74.98 ± 5.20^*∗*^	21.15 ± 2.32	32.74 ± 3.79^*∗*^	135.42 ± 7.49	194.77 ± 8.27^*∗*^
Control group (*n* = 53)	33.96 ± 3.37	47.58 ± 3.53^*∗*^	23.38 ± 2.68	29.91 ± 2.73^*∗*^	56.74 ± 4.49	67.51 ± 4.87^*∗*^	20.85 ± 3.50	28.40 ± 2.80^*∗*^	134.92 ± 7.76	173.66 ± 7.57^*∗*^
*t*	0.483	8.984	1.142	7.166	0.781	7.631	0.524	6.709	0.013	13.711
*P* value	0.574	0.000	0.256	0.000	0.437	0.000	0.602	0.000	0.990	0.000

*Note.* Compared with the group of before intervention, ^*∗*^*P* < 0.05.

## Data Availability

The data can be obtained from the corresponding author upon reasonable request.
